The article "Prevalence of p53 dysregulations in feline oral squamous cell carcinoma and non-neoplastic oral mucosa" was retracted in 2026. Reasons: duplicated images; overlap with earlier publications; concerns about the images; concerns about the results or conclusions.

# Prevalence of p53 dysregulations in feline oral squamous cell carcinoma and non-neoplastic oral mucosa

**DOI:** 10.1371/journal.pone.0215621

**Published:** 2019-04-18

**Authors:** Andrea Renzi, Paola De Bonis, Luca Morandi, Jacopo Lenzi, Debora Tinto, Antonella Rigillo, Giuliano Bettini, Emma Bellei, Silvia Sabattini

**Affiliations:** 1 Department of Veterinary Medical Sciences, University of Bologna, Ozzano Emilia, Bologna, Italy; 2 “M. Malpighi” Section of Anatomic Pathology, Department of Biomedical and Neuromotor Sciences, Bellaria Hospital, University of Bologna, Bologna, Italy; 3 Section of Hygiene, Public Health and Medical Statistics, Department of Biomedical and Neuromotor Sciences, University of Bologna, Bologna, Italy; Charles P. Darby Children’s Research Institute, 173 Ashley Avenue, Charleston, SC 29425, USA, UNITED STATES

## Abstract

Squamous cell carcinoma is the most common malignant oral tumor in cats. The late presentation is one of the factors contributing to the detrimental prognosis of this disease. The immunohistochemical expression of the p53 tumor suppressor protein has been reported in 24% to 65% of feline oral squamous cell carcinomas, but no study has systematically evaluated in this tumor the presence of p53 encoding gene (*TP53*) mutations. The aim of this retrospective study was to determine whether p53 immunohistochemistry accurately reflects the mutational status of the *TP53* gene in feline oral squamous cell carcinoma. Additionally, the prevalence of p53 dysregulation in feline oral squamous cell carcinoma was compared with that of feline non-neoplastic oral mucosa, in order to investigate the relevance of these dysregulations in cancer development. The association between p53 dysregulations and exposure to environmental tobacco smoke and tumor characteristics was further assessed.

Twenty-six incisional biopsies of oral squamous cell carcinomas and 10 cases each of lingual eosinophilic granuloma, chronic gingivostomatitis and normal oral mucosa were included in the study. Eighteen squamous cell carcinomas (69%) expressed p53 and 18 had mutations in exons 5–8 of *TP53*. The agreement between immunohistochemistry and mutation analysis was 77%. None of non-neoplastic oral mucosa samples had a positive immunohistochemical staining, while one case each of eosinophilic granuloma and chronic gingivostomatitis harbored *TP53* mutations. Unlike previously hypothesized, p53 dysregulations were not associated with exposure to environmental tobacco smoke. These results suggest an important role of p53 in feline oral tumorigenesis. Additionally, the immunohistochemical detection of p53 expression appears to reflect the presence of *TP53* mutations in the majority of cases. It remains to be determined if the screening for p53 dysregulations, alone or in association with other markers, can eventually contribute to the early detection of this devastating disease.

## Introduction

Squamous cell carcinoma is the most common malignant tumor of the oral cavity in cats, accounting for 60–70% of all oral malignancies. [1–3] Feline oral squamous cell carcinoma (FOSCC) most frequently involves the lingual region and dentate jaws, and may appear either as a necrotic ulcerative lesion or as a firm nodular swelling, generally associated with high local invasiveness and early bone lysis. [2, 3] Although regional and distant metastases have been reported, death most frequently occurs from complications associated with the primary tumor before metastatic disease has an opportunity to become clinically relevant. [3, 4–6] Due to location and rapid tumor progression, diagnosis is often late, and this largely limits the efficacy of treatments, including surgery, radiation therapy and chemotherapy. Prognosis is poor for the majority of cats, and, even with a multimodal therapeutic approach, the median survival time rarely exceeds 12 months. [2, 7, 8]

The p53 protein, encoded by the *TP53* oncosuppressor gene, counteracts the oncogenic transformation and tumor growth by preventing the replication of genetically damaged cells. [9, 10] Under unstressed physiologic conditions, the p53 protein has a half-life of 5–20 min in most cell types and is maintained at a low level, therefore it is normally not detected by immunohistochemical (IHC) methods [11]. Mutations of *TP53* may induce conformational changes that stabilize the protein, determining a nuclear accumulation of p53 that is detectable by IHC. [12–14]

Somatic mutations in the *TP53* gene are the most frequent alterations in human head and neck squamous cell carcinoma (HNSCC), detected in up to 85% of cases, and have been related to tobacco carcinogenesis. [15–17] In HNSCC, the IHC expression of p53 is also a frequent finding and has been historically considered an indirect evidence of mutations, although a disagreement between the two methods has been reported in up to 40% of cases. [18, 19]

In FOSCC, the IHC expression of p53 has been reported in 24% to 65% of cases, [20–22] and an association between p53 expression and exposure to household environmental tobacco smoke (ETS) was hypothesized. [21] Although an anecdotal report exists of a *TP53* mutation in a FOSCC, [23] no study has systematically evaluated the presence of *TP53* mutations in these tumors, nor their association with IHC protein expression. Understanding the mutational landscape of p53 in FOSCC may provide new insights to the molecular pathogenesis of this disease, and allow meaningful comparisons with human oral cancer.

The aim of this study was to determine whether p53 IHC accurately reflects the mutational status of the *TP53* gene in FOSCC, and to investigate the relationship between p53 dysregulations and ETS exposure in cats. Additionally, the prevalence of p53 expression and mutations in FOSCC was compared with feline normal oral mucosa and oral inflammatory lesions, in order to investigate the relevance of p53 dysregulation in cancer development.

## Materials and methods

### Ethics statement

This is a retrospective study on archived tissue samples of FOSCC. As the research did not influence any therapeutic decision, approval by an ethics committee was not required.

However, all diagnostic and therapeutic procedures were performed in accordance with the Public Health Service Policy on Humane Care and Use of Laboratory Animals.

All the examined samples were collected for diagnostic purposes as part of routine standard care. Owners gave informed consent to the use of clinical data and stored biological samples for teaching and research purposes.

### Case inclusion criteria and patient information

A retrospective survey was carried out on medical records of the Veterinary Hospital at the Department of Veterinary Medical Sciences (University of Bologna, Italy) from 2010 to 2018, in order to identify histologic samples of FOSCC and chronic oral inflammation. The histologic sections were microscopically reviewed to confirm the diagnosis. All consecutive cases of confirmed FOSCC were included, while 10 cases each of eosinophilic granuloma and chronic gingivostomatitis were selected. In addition, 10 post-mortem histologic samples of feline oral mucosa with normal histologic appearance were prospectively collected from cats with at least 7 years of age, deceased for causes unrelated to oral pathology. Samples were obtained from the maxillary premolar gum.

Patient records were reviewed to collect demographic information and tumor location. Cats’ owners were interviewed by e-mail or phone to collect information on ETS exposure, which was graded as follows: no exposure (owners not smoking indoors or cats living exclusively outdoors); mild exposure (1–5 cigarettes/day smoked indoors); moderate exposure (6–10 cigarettes/day smoked indoors); intense exposure (>10 cigarettes/day smoked indoors). The availability of this information was not among inclusion criteria.

### Histology

All samples for histological examination had been fixed in 10% neutral-buffered formalin, embedded in paraffin, sectioned at 4 μm and stained with hematoxylin and eosin (HE).

Histologic parameters evaluated for FOSCC included histologic subtype according to previously published criteria, [24, 25] histologic grade according to the Broders’ system (only for the conventional histotype), [26] and mitotic count (MC). MC was assessed as the total number of mitotic figures in a 2.37 mm^2^ area (10 fields with a 40x objective and a 10x ocular with a field number of 22 mm), according to the standards proposed by Meuten *et al*., 2016. [27] The count was performed in 10 consecutive non-overlapping high-power fields (HPFs), starting from an area of high mitotic activity. Fields with necrosis or inflammation were skipped. All histologic evaluations were performed by consensus by two of the authors (AR1 and PDB).

### Immunohistochemistry

Serial sections of FOSCC, eosinophilic granuloma, chronic gingivostomatitis and normal oral mucosa were immunolabeled for p53 using a commercial mouse monoclonal antibody (Pab 240 clone, BD Biosciences, San Jose, California, USA) with validated reactivity in feline tissues. [20, 22, 28]

Endogenous peroxidase activity was blocked by incubation for 10 min with 0.9% hydrogen peroxide in phosphate buffered saline (PBS, pH 7.2). For antigen retrieval, slides were microwaved in citrate buffer (pH 6.0) for 4 cycles of 5 min, at 750 W. After 4 washes of 5 min each with PBS containing 0.01% Tween 20 (p9416, Sigma Aldrich-Merck, Darmstadt, Germany) and 0.01% non-fat dry milk, slides were pre-incubated with 20% normal goat serum diluted in PBS containing 1% bovine serum albumin (BSA) for 20 min. Subsequently, slides were incubated in a humid chamber with the primary antibody diluted 1:100 in PBS containing 1% BSA for 80 min at room temperature. After another 4 washes of 5 min each with PBS containing 0.01% Tween 20 and 0.01% non-fat dry milk, binding sites of the primary antibody were identified using a biotinylated goat anti-mouse secondary antibody (Dako, Glostrup, Denmark) diluted 1:100 in PBS containing 1% BSA, for 30 min at room temperature. Sections were then incubated with a commercial streptavidin-biotin-peroxidase kit (Vectastain Elite ABC Kit, Vector Laboratories, Burlingame, CA, USA) and 3,3-diaminobenzidine (DAB tablets, Diagnostic BioSystems, Pleasanton, CA, USA) was used as chromogen. Counterstain was performed with Papanicolaou’s hematoxylin.

A p53 positive FOSCC was used as positive control for the primary antibody. Negative controls were obtained by omitting the primary antibody. Cases with at least 20% of p53-immunoreactive epithelial cells were considered positive, according to previous studies. [22, 28] Only nuclear staining was regarded as specific. Interpretation of the p53 IHC staining was performed by two of the authors (SS and AR2) without prior knowledge of *TP53* mutational status.

### *TP53* mutation analysis

Mutation analysis was performed at the “M. Malpighi” Section of Anatomic Pathology and at the Neurology Unit, IRCCS Institute of Neurological Sciences of Bologna, Department of Biomedical and Neuromotor Sciences, Bellaria Hospital, University of Bologna, Italy.

The *TP53* mutational status of each included case of FOSCC, inflammatory lesions and normal oral mucosa was assessed by deep sequence analysis of exons 5 through 8, corresponding to *TP53* DNA binding domain.

Primers and chromosome coordinates are detailed in Table 1. DNA from 10 μm sections of formalin-fixed and paraffin-embedded (FFPE) tissues (5 for each sample) was purified using the MasterPure Complete DNA extraction kit (Epicentre, code MC85200, Madison, WI, USA). If DNA amplification was not successful, the case was excluded from the study.

**Table 1:** *TP53* primers and coordinates.

Exons	Forward primer	Reverse primer	Genome coordinates
*TP53* exon 5	AGTACTCCCCTCCCCTCAAC	GCTCACCATCGCTACTGTCA	Chrom E1, strand -: 2451253–2451447 Amplicon length: 194 bp
*TP53* exon 6	ATTCCTCCCCGATTGCTCT	CTCCCAGAGACCCCAGATG	Chrom E1, strand -: 2451035–2451199 Amplicon length: 164 bp
*Tp53* exon 7	ACTCGGCCGGATCTTCTCT	CGGTAGCACGGGAGAGAGT	Chrom E1, strand -: 2450673–2450857 Amplicon length: 184 bp
*TP53* exon 8	TGCCTCCAGCTTCTGTCTTC	CTCCCTGCCTCYTCTCGTC	Chrom E1, strand -: 2450289–2450488 Amplicon length: 199 bp

Locus-specific amplicon libraries were generated with the application of tagged primers using multiplex PCR. The library preparation included two steps: a first PCR amplification for target enrichment, and a second shorter amplification session (8 cycles) to allow the barcoding of the template-specific amplicons obtained from the first amplification step. Barcoding was performed by using Nextera index kit as previously described. [29] Following each PCR step, the amplification products were purified using MagSi-NGSPREP (MagnaMedics, code MDKT00010075, Geleen Netherlands) and quantified with the Quantus Fluorometer (Promega, code E6150, Milan, Italy).

Sequencing was conducted on MiSeq sequencer (Illumina, San Diego, CA, USA), according to the manufacturer’s protocol.

Cases were classified as mutated when presenting one or more alterations in the nucleotide sequence of the amplified exons of feline *TP53*, resulting in amino acid changes with negative impact on the protein function according to PolyPhen-2, [30] and showing a variant allele frequency (VAF) >10%.

### Statistical analysis

Continuous data were tested for normality with the D’Agostino and Pearson omnibus normality test. Variables were summarized as mean ± standard deviation in case of normal distribution, or as median and range in case of non-normal distribution.

The agreement between p53 immunohistochemical expression and *TP53* mutation analysis was assessed using the Cohen’s kappa coefficient (*κ*). [31] Additionally, the relationship between p53 dysregulations (i.e., mutations or IHC expression) and the following variables was investigated: exposure to ETS (yes/no), diagnosis (FOSCC, chronic inflammatory lesions, normal oral mucosa), FOSCC location (dentate jaws, non-dentate mucosa, tongue), FOSCC histotype (conventional vs. non-conventional), conventional FOSCC degree of differentiation (well differentiated vs. moderately or poorly differentiated), and FOSCC MC. The distribution of categorical variables between groups was assessed using either the *χ*^*2*^ test or Fisher’s exact test; the distribution of quantitative variables between groups was assessed using either the unpaired two-sample *t*-test or Mann-Whitney *U* test. The choice between tests depended on the sample size and data distribution.

Analyses were carried out using a commercial software program (SPSS Statistics v19, IBM, Armonk, NY, USA); the significance level was set at 0.05.

## Results

The complete demographic, histological and molecular data of the cases in this study are provided in S1 and S2 Tables.

### FOSCC

Twenty-six incisional biopsies of FOSCC met the inclusion criteria. Breeds included 22 Domestic shorthair (DSH) cats, 2 Chartreux, one Siamese and one Persian. There were 12 castrated males and 14 spayed females. The median age was 14.5 years (range, 8–19). The information on ETS was available for 24 cats, 6 of which (25%) were exposed (mild exposure, n = 2; moderate exposure, n = 2; intense exposure, n = 2).

Tumors were located on mandibular gum (n = 12), maxillary gum (n = 6), tongue (n = 6), vestibular mucosa (n = 1) and hard palate (n = 1).

Twenty-two FOSCC (84%) belonged to the conventional histotype, 11 of them (50%) were well differentiated (grade 1 according to Broder’s grading system) and the remaining 11 were moderately differentiated (grades 2 and 3). Well differentiated FOSCC were characterized by neoplastic trabeculae with orderly progression from polyhedral, non-keratinized basal cells at the periphery to large, polygonal, keratinized cells with prominent intercellular bridges at the centers. Accumulations of amorphous to laminated keratin were frequently seen. Moderately differentiated FOSCC were characterized by disordered maturation, tumor cells with less eosinophilic cytoplasm and lack of evident intercellular bridges. Clusters of partially-keratinized cells were prevalent over keratin accumulation.

The remaining FOSCC belonged to the acantholytic (n = 2; 8%) and spindle cell (n = 2; 8%) histotypes.

The median MC was 13 in 10 HPF (range, 0–85).

Eighteen cases (69%) were positive for p53 IHC. The labelling was intense, with nuclear localization and was either visible in all neoplastic cells (n = 9; 34.6%) or confined to the periphery of the trabeculae (n = 9; 34.6%; Fig 1).

**Fig 1:** Cat, oral mucosa. Representative examples of p53 immunohistochemistry. (A) Squamous cell carcinoma. Intense nuclear labelling in all the neoplastic cells. (B) Squamous cell carcinoma. Intense nuclear labelling of the neoplastic cells at the periphery of the trabeculae (focal positivity). (C) Eosinophilic granuloma and (D) chronic gingivostomatitis. Moderate cytoplasmic staining of the inflammatory cells. (E) Chronic gingivostomatitis. Weak staining in less than 20% of nuclei in the basal and suprabasal layers of the epithelium, which appears moderately hyperplastic. (F) Normal oral mucosa. Lack of positive staining. 200x magnification. Haematoxylin counterstain.

Nineteen mutations of *TP53* were detected in 18 cases (69%); there were 16 missense mutations, 1 nonsense mutation and 2 in frame deletions; all the examined exons were involved (exon 5, n = 6; exon 6, n = 3; exon 7, n = 6; exon 8, n = 4).

Of the 18 FOSCC with IHC p53 expression, 3 cases with focal immunolabeling did not harbor *TP53* mutations. Of the 18 tumors with mutated *TP53*, 3 were p53-negative; among these, case 10 showed a PolyPhen2 score of 0.756, indicating only a possible damage; case 13 showed two mutations both with a PolyPhen2 score of 1.00, indicating full protein damage, with a 60% and 27% VAF for p.Y155* and p.R206Q respectively. Finally, case 6 showed a single point mutation in codon 207 (p.H207P) with a VAF of 13% and PolyPhen2 sore of 1.00; S1 Table). Overall, there was agreement in 77% of FOSCC. The *κ* coefficient was 0.46 (*P* = 0.010), indicating a moderate agreement between p53 immunohistochemical expression and *TP53* mutation analysis.

### Chronic inflammatory lesions

Cases of eosinophilic granuloma belonged to 10 DSH cats, 5 castrated males (50%) and 5 spayed females (50%). The median age was 9 years (range, 1–14). All lesions were located on the tongue (dorsal aspect, n = 5; ventral aspect/frenulum, n = 4; lateral margin, n = 1).

Cats with chronic gingivostomatitis were 9 DSH and one Maine Coon; 7 (70%) were castrated males and 3 (30%) spayed females. The median age was 11.5 years (range, 1–15). All lesions were located on the dentate jaws (maxillary gum, n = 5; mandibular gum, n = 5).

The information on ETS was available for 16 out of 20 cats, 4 of which (25%; eosinophilic granuloma, n = 2; chronic gingivostomatitis, n = 2) were exposed (mild exposure, n = 1; moderate exposure, n = 1; intense exposure, n = 2).

Histologically, eosinophilic granulomas were characterized by a subepithelial infiltrate of eosinophils and mononuclear cells, with the presence of "flame figures", consisting of deposits of amorphous eosinophilic material surrounded by macrophages and multinucleated giant cells. In chronic gingivostomatitis, the corium was expanded by variable amounts of lymphocytes and plasma cells, and covered by ulcerated to hyperplastic epithelium.

All inflammatory lesions were negative for p53 IHC, although showing a weak staining in < 20% of epithelial cells, predominantly located in the basal layer of the hyperplastic areas. A weak cytoplasmic staining was also observed in the subepithelial stroma, endothelial cells and inflammatory cells.

*TP53* missense mutations were detected in one eosinophilic granuloma (10%) and one chronic gingivostomatitis (10%); mutations were located in exons 5 (n = 1), 6 (n = 1) and 7 (n = 2; S2 Table).

### Normal oral mucosa

The 10 normal oral mucosa samples belonged to 9 DSH and 1 Chartreux; 7 males (70%; 6 castrated) and 3 spayed females (30%). The median age was 11 (range, 7–17). The causes of death included cardiomyopathy (n = 3), chronic kidney disease (n = 2), intestinal lymphoma (n = 2), hemorrhagic cystitis (n = 1), pulmonary carcinoma (n = 1), and meningioma (n = 1).

Three cats (30%) were exposed to ETS (mild exposure, n = 2; moderate exposure, n = 1).

None of the samples was positive for p53 IHC, and no *TP53* mutation was detected (S2 Table).

### Statistical analysis of p53 dysregulations

Overall, the agreement between p53 immunohistochemistry and mutation analysis was 86%.

The κ coefficient was 0.68 (P < 0.001), indicating a substantial agreement between p53 immunohistochemical expression and *TP53* mutation analysis. Both p53 IHC overexpression and *TP53* mutations were significantly more frequent in FOSCC, and mutated cases had a significantly lower MC (Tables 2 and 3). There was no statistical relationship between p53 dysregulations and the other evaluated variables, including exposure to ETS (Tables 2 and 3).

**Table 2:** Relationship between p53 immunohistochemical expression and other clinicopathological variables in 56 histological samples of feline oral mucosa.

Variable	p53 not expressed	p53 expressed	P
**ETS** (n = 50)	(4 missing)	(2 missing)	0.508
exposed	10 (29%)	3 (19%)	
not exposed	24 (71%)	13 (81%)	
**Diagnosis** (n = 56)			<0.001
FOSCC	8 (21%)	18 (100%)	
chronic inflammatory lesions	20 (53%)	0 (0%)	
normal oral mucosa	10 (26%)	0 (0%)	
**FOSCC location** (n = 26)			0.657
dentate jaws	6 (75%)	12 (67%)	
non-dentate mucosa	1 (13%)	1 (6%)	
tongue	1 (13%)	5 (28%)	
**FOSCC histotype** (n = 26)			0.563
conventional	6 (75%)	16 (89%)	
non conventional	2 (25%)	2 (11%)	
**Conventional FOSCC degree of differentiation** (n = 22)			0.635
well differentiated	2 (33%)	9 (56%)	
moderately/poorly differentiated	4 (67%)	7 (44%)	
**FOSCC MC** (n = 26) (median, range)	16 [6–85]	11 [0–81]	0.388

Abbreviations: ETS, environmental tobacco smoke; FOSCC, feline oral squamous cell carcinoma; MC, mitotic count.

**Table 3:** Relationship between *TP53* mutations and other clinicopathological variables in 56 histological samples of feline oral mucosa.

Variable	*TP53* wild-type	*TP53* mutated	*P*
**ETS** (n = 50)	(3 missing)	(3 missing)	>0.999
exposed	9 (27%)	4 (24%)	
not exposed	24 (73%)	13 (76%)	
**Diagnosis** (n = 56)			<0.001
FOSCC	8 (22%)	18 (90%)	
chronic inflammatory lesions	18 (50%)	2 (10%)	
normal oral mucosa	10 (28%)	0 (0%)	
**FOSCC location** (n = 26)			0.283
dentate jaws	4 (50%)	14 (78%)	
non-dentate mucosa	1 (13%)	1 (6%)	
tongue	3 (38%)	3 (17%)	
**FOSCC histotype** (n = 26)			0.563
conventional	6 (75%)	16 (89%)	
non conventional	2 (25%)	2 (11%)	
**Conventional FOSCC degree of differentiation** (n = 22)			0.635
well differentiated	2 (33%)	9 (56%)	
moderately or poorly differentiated	4 (67%)	7 (44%)	
**FOSCC MC** (n = 26) (median, range)	16.5 [10–85]	7.5 [0–79]	0.034

Abbreviations: ETS, environmental tobacco smoke; FOSCC, feline oral squamous cell carcinoma; MC, mitotic count.

## Discussion

There are many similarities at both clinical and molecular level between HNSCC and FOSCC, which has led to the proposal that FOSCC may serve as a spontaneous model for human disease. [22, 32, 33]

Herein, we provide further evidence to this hypothesis, by demonstrating in FOSCC a high prevalence (69%) of mutations in the DNA binding domain of *TP53*. This is also the most frequent site of somatic genomic alterations in HNSCC, and the most important region for folding and stabilization of the tertiary structure of the protein, suggesting the importance of the loss of function of the p53 pathway in the development and progression of oral cancer in both species. [19, 34]

While cells with functional p53 respond to DNA damage by undergoing cell-cycle arrest, DNA repair or apoptosis, cells lacking functional p53 may continue to divide and accumulate genetic damages, thus leading to a potential malignant transformation. Although p53 mutants can be classified by their effect on protein structure, it is currently not possible to predict precisely how a particular mutation impairs function [34].

In most cases, mutations were also associated with p53 IHC expression, as confirmed by an agreement of 77%. Predictably, discordant results were obtained, including 3 IHC positive cases with no *TP53* mutation and 3 IHC negative cases harboring *TP53* mutations. In humans, positive results in p53 IHC have formerly been interpreted as indicating inactivation of the *TP53* gene, based on the knowledge that the half-life of the wild-type protein is too short to permit detection, whereas the mutant protein is more stable. However, the role of p53 immunostaining as a surrogate marker of *TP53* gene alterations has been downgraded over time. [19, 35] Although IHC is rapid, relatively inexpensive, and widely available to most diagnostic laboratories, a number of biological and technical factors may contribute to limit its correlation with genetic analysis. p53 expression in the absence of detectable mutations may be related to the presence of genetic alterations outside the DNA binding domain; alternatively, post-transcriptional protein accumulation may result from aberrant degradation or induction by genotoxic insults; whereas stabilization can be mediated by cellular and transforming viral proteins. [19, 36, 37] In humans, papillomavirus (PV) E6 protein may produce a similar effect; however, while PV DNA sequences have been detected in a small proportion of FOSCC, there is currently no evidence that PV has a role in the development of oral cancer in cats. [38]

Absence of IHC positivity in mutated FOSCC could be due to mutations that do not result in protein stabilization, undetectable truncated proteins or deletions that inhibit transcription altogether. Furthermore, mutations which render a conformational change not recognized by the primary antibody will generate false negatives, as may result for cases 6, 10, and 13. [35, 39] In case 13 the simultaneous presence of two damaging mutations (p.Y155*; p.R206Q) with high VAF and high Polyphen2 score may justify the loss of p53 staining. The same immunostaining behavior was detected for case 6, harboring a damaging mutation in p.H207P, very close to p.R206Q. The low VAF (13%) and probably the region involved may be the cause of undetectable IHC signal. Finally, case 10 showed a Polyphen2 score of 0.756, indicating only a possible protein damage, probably not enough to be recognized by the p53 Pab 240 clone.

In addition to these biological mechanisms, technical limitations may also give account for discrepancies between p53 IHC and mutational analysis, including the choice of the antibody and of the thresholds for positive p53 staining and variant allele frequency. [36] Numerous monoclonal antibodies are available for the IHC analysis of human p53 protein, and the sensitivity of the immunostaining can be refined by using different clones simultaneously. Currently, the p53 antibodies with known immunoreactivity in feline tissues are PAb240 and CM-1. A study on different canine neoplasms obtained the highest percentage of positive cases with the polyclonal antibody CM-1; [40] nevertheless, in this study the PAb 240 clone was preferred, because it has been reported to produce less background staining than CM-1 and to recognize more specifically the mutant epitopes of p53. [20, 22, 28, 40, 41] Additional technical issues may relate to the formalin fixation process, which on the one hand might limit the immunoreactivity of samples and on the other hand induce excessive DNA fragmentation.

This study reports a significantly higher prevalence of p53 dysregulation in FOSCC compared with non-neoplastic oral lesions, further supporting a role of p53 in oral tumorigenesis. This apparent specificity also makes p53 a potential candidate for investigation as a diagnostic biomarker. In humans, p53 mutations are important determinants of the malignant potential of oral lesions and have been detected in the saliva and blood of HNSCC-bearing patients. [19, 42, 43] In cats, no oral lesions of confirmed or presumed preneoplastic significance have so far been identified, and early neoplastic disease may be hard to differentiate from other chronic inflammatory or proliferative lesion of the oral mucosa. Dental disease with associated periodontitis, gingivitis and gingival hyperplasia is a common finding in elderly cats, and idiopathic ulcerative lesions belonging to the feline eosinophilic granuloma complex and mimicking FOSCC may occur on the tongue or frenulum. [3] Even histologically, the early distinction between neoplastic and inflammatory disorders can be challenging: squamous cell carcinomas are frequently accompanied by an inflammatory response, due to the presence of epithelial ulceration and keratin production. In turn, chronic stomatitis may induce hyperplastic-dysplastic changes of the mucosa that can hardly be differentiated from early neoplastic transformation.

Since the early detection of FOSCC is the only weapon currently available to effectively fight this disease, further studies are worth to assess the diagnostic potential of p53, alone or in association with other molecular markers. In this scenario, it is interesting to speculate whether the two mutations with no concurrent IHC expression found in inflammatory lesions should be regarded as nonspecific findings or as the result of an early inflammation-driven carcinogenesis. Considering the frequency of chronic stomatitis in geriatric cats, it can be difficult to estimate how reliable is the risk of a neoplastic transformation of these lesions.

The pathogenesis of FOSCC is not well characterized, but exposure to tobacco smoke has been postulated as a potential risk factor, among others, potentially due to the grooming habits of cats increasing the oral dose of environmental carcinogens. [44] Furthermore, in one study, tumors from cats exposed to ETS were 4.5 times more likely to overexpress p53 than were tumors from unexposed cats, although this association was not statistically significant. [21] In the present study, exposure to tobacco smoke was unfrequently observed in cats with SCC, being reported in 6 out of 24 cases, and was not associated with either p53 expression or *TP53* mutations. While not excluding the carcinogenetic effect of ETS in FOSCC, these results let us hypothesize that other factors may have triggered the dysregulation of the p53 pathway in these cats.

The main limits of this study are the small number of cases and its retrospective design, with consequent lack of standardized therapy protocols. This also impairs any consideration on the biologic behavior of mutated tumors and, ultimately, on the prognostic significance of p53.

## Conclusions

These results suggest an important role of p53 in feline oral tumorigenesis. This is supported by a significantly higher prevalence of p53 dysregulation in FOSCC compared with normal oral mucosa and inflammatory lesions. Additionally, the IHC detection of p53 expression appears to reflect the presence of p53 mutations in the majority of cases. It remains to be determined if the screening for p53 dysregulations, alone or in association with other markers, may contribute to the early detection of this detrimental disease, and eventually help to make it more curable.

## Supporting information

S1 Table Demographic, histological and molecular data of 26 cases of feline oral squamous cell carcinoma. (XLSX)

S2 Table Demographic, histological and molecular data of 30 cases of non-neoplastic feline oral mucosa. (XLSX)
